RETRACTED

# Mesenteric Panniculitis and COVID-19: A Rare Association

**DOI:** 10.7759/cureus.21314

**Published:** 2022-01-17

**Authors:** Israa A Alyousef, Zainab A Alsaileek, Manar A Alabdulsalam, Muhannad A Almohanna, Naif A Alshaqhaa, Mohammed M Alqahtani, Anas A Al Alyany, Muhannad A Alzahrani, Hawazin A Fallatah, Jalal I Alqadhib, Abdulaziz M Alhawsawi, Abdulelah D Alsuhaymi, Ali M Alasmari, Abdullah J Alshareef, Faisal Al-Hawaj

**Affiliations:** 1 College of Medicine, Dar Al Uloom University, Riyadh, SAU; 2 College of Medicine, Qassim University, Buraydah, SAU; 3 College of Medicine, Almaarefa University, Riyadh, SAU; 4 College of Medicine, Jordan University of Science and Technology, Irbid, JOR; 5 College of Medicine, Al-Baha University, Al-Baha, SAU; 6 College of Medicine, King Abdulaziz University, Jeddah, SAU; 7 College of Dentistry, Imam Abdulrahman Bin Faisal University, Dammam, SAU; 8 General Practice, Madinah General Hospital, Medina, SAU; 9 College of Medicine, Hunan Normal University, Changsha, CHN; 10 College of Medicine, Umm Al-Qura University, Mecca, SAU; 11 College of Medicine, Taif University, Taif, SAU; 12 College of Medicine, Imam Abdulrahman Bin Faisal University, Dammam, SAU

**Keywords:** computed tomography, case report, mesenteric panniculitis, abdominal pain, covid-19

## Abstract

Coronavirus disease 2019 (COVID-19) typically involves the respiratory system, but gastrointestinal involvement is common. Further, patients with severe COVID-19 are at high risk to develop gastrointestinal complications, including bowel ischemia, ileus, and deranged liver enzymes. We present the case of a 44-year-old woman with mild COVID-19 pneumonia who was in home isolation. Ten days after the isolation, the patient presented to the emergency department complaining of generalized abdominal pain that was sharp in nature and associated with nausea and recurrent episodes of vomiting. The patient did not complain of any respiratory symptoms. Physical examination showed diffuse tenderness with no clinical signs to suggest generalized peritonitis. The laboratory parameters showed normal hematological, renal, and hepatic profiles. No elevation in the inflammatory markers was observed. The amylase level was within the normal range. Abdominal computed tomography scan demonstrated the presence of misty mesentery with increased density of the mesentery with fat stranding encasing the mesenteric vessels along with mesenteric adenopathy. Such radiological features suggested the diagnosis of mesenteric panniculitis. Subsequently, intravenous corticosteroid therapy was initiated and the patient exhibited significant improvement after 24 hours. The patient was discharged after nine days of hospitalization. She was followed up after one month and she had no complaints. Mesenteric panniculitis is a rare idiopathic inflammatory condition involving the mesenteric adipose tissue. The case shed a light on the possible association of COVID-19 with mesenteric panniculitis. The clinical manifestations of mesenteric panniculitis are non-specific and imaging studies are essential to suggest the diagnosis.

RETRACTED

## Introduction

Coronavirus disease 2019 (COVID-19) typically involves the respiratory system and manifests with fever, dyspnea, and cough. However, gastrointestinal symptoms in COVID-19 are common. It is reported that over 50% of patients reported at least one gastrointestinal symptom in addition to respiratory complaints [1]. Further, some reports suggested that the gastrointestinal symptoms may indeed precede the respiratory manifestations of COVID-19 [2]. Patients with COVID-19 who present with gastrointestinal symptoms tend to have a milder course of the disease [3]. However, patients with severe COVID-19 are at high risk to develop gastrointestinal complications, including bowel ischemia, ileus, and deranged liver enzymes [4]. A retrospective study by Giraudo et al. [5] involving 113 computed tomography scans of patients with confirmed COVID-19 pneumonia revealed that 13% of patients had increased attenuation of the mesenteric fat giving the appearance of “misty mesentery”. Here, we report the case of a patient on home isolation after COVID-19 pneumonia who developed acute abdominal pain due to mesenteric panniculitis.

## Case presentation

A 44-year-old woman presented to the emergency department with a history of cough and fever for four days. The cough was not productive of sputum. The fever was constant and measured 38.1℃ in its peak. It was resolved by the use of oral paracetamol. Her symptoms were not associated with chest pain or dyspnea. She was otherwise healthy with no history of comorbid conditions. She was a non-smoker. The family and social history were non-contributory. The physical examination revealed normal oxygen saturation on room air with normal vital signs, including the pulse rate and respiratory rate. The patient had a body mass index of 28 kg/m^2^ (height 159 cm, weight 71 kg). Scattered crepitations were noted throughout both lung fields.

The patient underwent a reverse-transcriptase polymerase chain reaction test that was positive for the severe acute respiratory syndrome coronavirus 2 (SARS-CoV-2). Since the patient’s symptoms were mild and she had no previous comorbid conditions, she was offered the option to have home isolation according to the national protocol.

Ten days later, the patient presented to the emergency department complaining of generalized abdominal pain that was sharp in nature and associated with nausea and recurrent episodes of vomiting. The patient did not complain of any respiratory symptoms. Physical examination showed diffuse tenderness with no clinical signs to suggest generalized peritonitis. The laboratory parameters showed normal hematological, renal, and hepatic profiles. No elevation in the inflammatory markers was observed on the initial and subsequent tests. The amylase level was within the normal range. The coagulation profile was normal.

RETRACTED

The general surgery team was consulted and advised for an abdominal computed tomography scan. Subsequently, the contrast-enhanced computed tomography demonstrated the presence of misty mesentery with increased density of the mesentery with fat stranding encasing the mesenteric vessels along with mesenteric adenopathy (Figures 1, 2). Such radiological features suggested the diagnosis of mesenteric panniculitis.

**Figure 1:** Axial CT image shows increased attenuation of the mesenteric fat. CT: computed tomography

**Figure 2:** Coronal CT image shows misty mesentery with increased density of the mesentery with fat stranding encasing the mesenteric vessels. CT: computed tomography

Subsequently, intravenous corticosteroid therapy (intravenous methylprednisolone 40 mg) was initiated to prevent the progression of the disease and the fibrotic changes. The patient exhibited significant improvement in her symptoms after 24 hours from the treatment. The steroid therapy was continued for seven days with tapering down the dose. The patient was discharged after nine days of hospitalization. She was followed up after one month and she had no complaints.

## Discussion

Mesenteric panniculitis is a rare benign non-specific inflammatory condition involving the intestinal mesentery. Mesenteric panniculitis is a rare condition with an average age of presentation in the seventh decade of life. It is twice as common in men as in women [6]. Considering the rarity of mesenteric panniculitis, its natural history is incompletely understood. The rate and risk factors of progression to the chronic stage are unknown. In the present case, since the patient had complete resolution of her symptoms, no further radiologic follow-up was performed to identify the presence of fibrosis changes.

The exact pathogenesis of mesenteric panniculitis remains unknown. However, several theories have been suggested. It is thought that mesenteric panniculitis develops as an inflammatory reaction following a prior abdominal surgery or trauma. This theory is supported by the finding of a cohort study showing that over 80% of patients with mesenteric panniculitis had a history of previous abdominal surgery [7]. Further, it has been suggested that a mesenteric panniculitis is a form of autoimmune condition targeting the adipose tissue of the mesentery. This is supported by the finding that some patients with mesenteric panniculitis have concomitant autoimmune disorders such as retroperitoneal fibrosis and primary sclerosing cholangitis. Additionally, mesenteric panniculitis can be a manifestation of paraneoplastic syndrome due to underlying malignancy [8,9]. However, in the present case, the patient had no history of any such risk factors, making the association between the panniculitis and COVID-19 more plausible. The SARS-CoV-2 virus uses the angiotensin-converting enzyme 2 (ACE2) as a receptor to invade human cells. Tissues with greater expression of ACE2 may become a target for the SARS-CoV-2. In addition to lung, the ACE2 is expressed in adipose tissue. Furthermore, it has been suggested that the expression of ACE2 in adipose tissue is higher than that in the lung tissue [10].

RETRACTED

The majority of patients with mesenteric panniculitis have no clinical symptoms and their disease is diagnosed incidentally on imaging studies performed for unrelated indications [9]. Symptomatic patients have abdominal pain that could be associated with fever, nausea, vomiting, and weight loss [6]. In the chronic fibrosis stage of the disease, patients may present with intestinal obstruction. The laboratory markers may show elevation of the C-reactive protein to suggest an underlying inflammatory process [8]. However, laboratory investigation findings are non-specific and may be normal as in the present case. Patients should be started with immunosuppressive therapy with corticosteroid being the first-line regimen. Other agents include cyclophosphamide, which can be attempted if no clinical improvement was noted with the corticosteroid therapy. Surgery has a limited role such as a palliative procedure to relieve bowel obstruction [6,9].

## Conclusions

Mesenteric panniculitis is a rare idiopathic inflammatory condition involving the mesenteric adipose tissue. The case shed a light on the possible association of COVID-19 with mesenteric panniculitis. The clinical manifestations of mesenteric panniculitis are non-specific and imaging studies are essential to suggest the diagnosis. Once the diagnosis is made, patients should be started on immunosuppressive therapy in order to prevent the chronic fibrotic changes of the disease.
